RETRACTED

# Design Computer-Aided Diagnosis System Based on Chest CT Evaluation of Pulmonary Nodules

**DOI:** 10.1155/2022/7729524

**Published:** 2022-01-10

**Authors:** Hui Wang, Yanying Li, Shanshan Liu, Xianwen Yue

**Affiliations:** ^1^Department of Radiology, The Second Affiliated Hospital of Harbin Medical University, 150086 Harbin, Heilongjiang, China; ^2^Department of Radiology, Weifang Respiratory Disease Hospital, Weifang, 261041 Shandong, China

## Abstract

At present, the diagnosis and treatment of lung cancer have always been one of the research hotspots in the medical field. Early diagnosis and treatment of this disease are necessary means to improve the survival rate of lung cancer patients and reduce their mortality. The introduction of computer-aided diagnosis technology can easily, quickly, and accurately identify the lung nodule area as an imaging feature of early lung cancer for the clinical diagnosis of lung cancer and is helpful for the quantitative analysis of the characteristics of lung nodules and is useful for distinguishing benign and malignant lung nodules. Growth provides an objective diagnostic reference standard. This paper studies ITK and VTK toolkits and builds a system platform with MFC. By studying the process of doctors diagnosing lung nodules, the whole system is divided into seven modules: suspected lung shadow detection, image display and image annotation, and interaction. The system passes through the entire lung nodule auxiliary diagnosis process and obtains the number of nodules, the number of malignant nodules, and the number of false positives in each set of lung CT images to analyze the performance of the auxiliary diagnosis system. In this paper, a lung region segmentation method is proposed, which makes use of the obvious differences between the lung parenchyma and other human tissues connected with it, as well as the position relationship and shape characteristics of each human tissue in the image. Experiments are carried out to solve the problems of lung boundary, inaccurate segmentation of lung wall, and depression caused by noise and pleural nodule adhesion. Experiments show that there are 2316 CT images in 8 sets of images of different patients, and the number of nodules is 56. A total of 49 nodules were detected by the system, 7 were missed, and the detection rate was 87.5%. A total of 64 false-positive nodules were detected, with an average of 8 per set of images. This shows that the system is effective for CT images of different devices, pixel pitch, and slice pitch and has high sensitivity, which can provide doctors with good advice.

## 1. Introduction

Pulmonary nodules are one of the most important clinical manifestations of early lung cancer. Only by fully understanding the characteristics of nodules and correctly diagnosing such nodules, patients with malignant nodules can receive functional treatment in time and avoid unnecessary surgery. Computer-aided diagnosis of benign and malignant pulmonary nodules is very important in clinic. Most of the early stage lung cancer is mainly assisted in diagnosis by computer tomography imaging technology. The imaging principle of CT is established based on the detection of the corresponding absorption degree of the radiation reflected by the tissues of different densities in patient's human body. The advantages of CT diagnosis are convenient and rapid examination, high-density resolution, quantitative measurement of CT value of tissue, clear CT image, and clear anatomical relationship. The disadvantage is that CT diagnosis has certain radiation, and there are still great limitations in the diagnostic efficiency of soft tissue tumors, especially in qualitative diagnosis. CT imaging overcomes the defects of traditional X-ray plain film image overlap and little difference in the density of adjacent organs and cannot form a contrast picture, and soft arrangement organs cannot develop or develop poorly. Specifically, after the radiation penetrates the human body, due to a certain attenuation law, the detector measures the attenuation of the radiation intensity, which is equivalent to the different absorption coefficients present on the tested plane. The numerical distribution of these absorption coefficients on the grid array is the image data. With the rapid development of medical imaging technology, CT technology has greatly improved its temporal and spatial resolution characteristics. Computed tomography (CT) and magnetic resonance (MRI) have different indications due to their different imaging principles. (CT) examination is an X-ray examination. It can scan all organs of the whole body. The scanning speed is fast. In a few seconds or more, an organ or whole body can be examined. Nuclear magnetic resonance (MRI) is a safer examination using magnetic field and radio pulse imaging, which is suitable for any population, including children and pregnant women. However, the application of MRI was limited in the past, mainly due to the slow scanning speed. Now, it is changed to a fully digital MRI equipment, and the scanning time is faster and faster, which benefits patients a lot. The resulting images can easily detect lesions with a diameter range of less than 1 mm.

RETRACTED

However, the current CT imaging technology can adjust the slice thickness of the image to be as thin as possible according to the needs of the specific application, which results in a huge volume of CT images of the lungs in each case, and sometimes, the number of slices is even as high as hundreds of slices. Faced with a large amount of image information and data every day, clinical scientists are sometimes inaccurate in traditional medical examination. The introduction of computer-aided diagnosis technology is of great significance. It can not only improve the diagnosis level and reduce unnecessary time but also locate the area of pulmonary nodules. At the same time, it can also quantitatively analyze the characteristics of pulmonary nodules, so as to provide diagnostic procedures for doctors to judge the benign and malignant degree of pulmonary nodules. At present, most CT scanning methods used in clinic include three kinds: localization image scanning mode, axial scan mode, and spiral scan.

Computer-aided diagnosis is developing rapidly. Computers have enabled radiologists and related experts at home and abroad to apply and process data more effectively and to detect and quantify lesions more effectively. Computer assistance is of great value in identifying previously overlooked information and reducing false positives. Han et al. proposed a computer-aided automatic diagnosis system for lung cancer, which can detect lung nodules early from the spiral CT images of the chest. The diagnostic system designed by it includes analysis and diagnostic procedures. In the analysis process, fuzzy clustering algorithm is first used to extract lung and pulmonary blood vessel regions, and then, image processing technology is used to analyze the characteristics of these regions. In the diagnosis process, we use the extracted features to define the diagnosis rules, and these features support the determination of candidate nodule positions. By applying the results of its application to image data for large-scale screening of 450 patients, we have demonstrated the effectiveness of the system. But the experiment is not very convincing [1]. Jin et al. have developed a computer-aided diagnosis (CAD) system that uses a 3D AC model based on two-dimensional AC and adds three new energy components to use 3D information. The volume of lung nodules segmented by the 3DAC model is used to achieve the best classification, which is usually better than that obtained by LIDC radiologists based on the visual judgment of the nodule boundary. The volume of lung nodules is large, but the experimental results are not very accurate [2]. The texture features of Xie et al. chest CT images used in the evaluation of malignant lung nodules have become a nonnegligible and effective factor in computer-aided diagnosis. Focus on extracting as few effective texture features as possible, which can be combined with other classic features to assist in the diagnosis of lung nodules. The experiment proved that the two extracted 3D Haralick projection features may help to classify benign and malignant nodules. However, the experiment did not take into account factors such as the thickness of lung nodules, which has certain limitations [3].

RETRACTED

This paper mainly studies the pulmonary nodule diagnosis system based on CT image and designs and implements it. It can be used in all parts of the body, including the head, neck, facial features, chest, abdomen, pelvic cavity, spine, and limbs. Theoretically, all lesions with changes in lesion density or morphology are suitable for CT examination, including tumors such as lung cancer and liver cancer. The main innovations are as follows: (1) lung region extraction is an important preprocessing step for automatic detection of lung nodules. The results of lung region segmentation in the experiment will directly affect the efficiency and effect of lung nodule detection algorithm. (2) The lung region segmentation method proposed in this paper makes use of the obvious differences between the lung parenchyma and other human tissues connected with it, as well as the position relationship and shape characteristics of each human tissue in the image. For the lung boundary caused by noise and pleural nodule adhesion, the segmentation of lung wall is inaccurate, and there is a problem of depression. (3) A multiscale relative convex hull technique is proposed to detect the concave surface of lung boundary.

## 2. Design of Auxiliary Diagnosis System for Chest CT Assessment of Pulmonary Nodules

### 2.1. Implementation of Lung Parenchymal Segmentation Algorithm

The basic process framework of lung parenchymal segmentation is roughly divided into three parts: binarization processing, lung parenchymal extraction, left and right separation of lung parenchyma, and edge repair.

1. Binarization of adaptive threshold

Threshold method is the most commonly used method of lung parenchymal segmentation. As shown in Figure 1, the lung parenchyma in the chest CT image can essentially be regarded as an air sac. The lungs are filled with air. The CT image is characterized as a dark area (corresponding to the low-density main peak area on the left in the gray-scale histogram). And there is a sharp contrast between muscles, vertebrae, ribs, and other tissues in the adjacent thoracic cavity (corresponding to the high-density double-peak area on the right in the gray-scale histogram). If a suitable threshold can be found between these two density areas with thresholding, the image can be binarized to separate the target from the background [4, 5]. Therefore, the threshold method is suitable for rough image segmentation.

RETRACTED

However, under special physiological and pathological conditions, the image information will be different. In this case, the fixed threshold method may cause segmentation failure. Therefore, a method of calculating the threshold based on the statistical characteristics of the image is selected to solve the above problems, and it has a certain degree of adaptability. The maximum between-class variance threshold method (Otsu method) is an adaptive unsupervised rule classification method [6, 7]. When the probability distribution of the overall gray-scale feature of the image is known, the threshold is determined according to the maximum value of the distance between classes. The specific principles are as follows.

Suppose there are *N* pixels in the image, among the *L* gray levels, the number of pixels with the gray value *i* is *n*_*i*_(0 ≤ *i* ≤ *L* − 1) and *N* = ∑_*i*=0_^*L*−1^*n*_*i*_. Therefore, the probability of each gray value is:

(1) $$\begin{array}{c} p_{i}=\frac{n_{i}}{N},0\leq p_{i}\leq 1,\overset{L-1}{\underset{i=0}{\sum }}p_{i}=1. \end{array}$$

Use *t* to represent the threshold value, then the background class and target class are, respectively, expressed as:

(2) $$\begin{array}{c} p_{1}=\overset{t}{\underset{i=0}{\sum }}\frac{n_{i}}{N},p_{2}=\overset{t}{\underset{i=t+1}{\sum }}\frac{n_{i}}{N},p_{1}+p_{2}=1. \end{array}$$

And their gray mean values are:

(3) $$\begin{array}{c} \mu_{1}=\overset{t}{\underset{i=0}{\sum }}\frac{{ip}_{i}}{p_{1}},\mu_{2}=\overset{L-1}{\underset{i=t+1}{\sum }}\frac{{ip}_{i}}{p_{2}}. \end{array}$$

The average gray level of the image is:

(4) $$\begin{array}{c} \mu_{0}=p_{1}\mu_{1}+p_{2}\mu_{2}=\overset{L-1}{\underset{i=0}{\sum }}{ip}_{i}. \end{array}$$

The between-class variance is defined as:

(5) $$\begin{array}{c} \sigma_{B}^{2}=p_{1}{\left(\mu_{1}-\mu_{0}\right)}^{2}+p_{2}{\left(\mu_{2}-\mu_{0}\right)}^{2}. \end{array}$$

In order to get the best threshold *t*^∗^ is to require the largest between-class variance:

(6) $$\begin{array}{c} t^{*}=\arg\underset{0\leq t\leq L-1}{\max}\left\{p_{1}{\left(\mu_{1}-\mu_{0}\right)}^{2}+p_{2}{\left(\mu_{2}-\mu_{0}\right)}^{2}\right\}. \end{array}$$

Considering *μ*_0_ = *p*_1_*μ*_1_ + *p*_2_*μ*_2_ and *p*_1_(*μ*_1_ − *μ*_0_)^2^ + *p*_2_(*μ*_2_ − *μ*_0_)^2^ = (*μ*_1_ − *μ*_0_)(*μ*_2_ − *μ*_0_), according to Equation (6), we can get:

(7) $$\begin{array}{c} t^{*}=\arg\underset{0\leq t\leq L-1}{\max}\left\{\left(\mu_{1}-\mu_{0}\right)\left(\mu_{2}-\mu_{0}\right)\right\}. \end{array}$$

Although Equation (6) and Equation (7) are equivalent, when the algorithm is implemented, comparing the two before and after, it is obvious that the algorithm complexity of the latter is relatively simple, and only the average value is solved, and the traversal space is reduced during the solution process, which has better timeliness [8, 9]. The optimal threshold *t*^∗^ constructs the rule classifier *g*(*x*), and its functional relationship is shown

(8) $$\begin{array}{c} g\left(x\right)=\left\{\begin{array}{cc} 1, & \left(x\leq t^{*}\right),\\ 0, & \left(x>t^{*}\right). \end{array}\right. \end{array}$$

As shown in Figure 2, the classifier is the core component in the binarization process, and the selection of the threshold directly affects the segmentation performance.

(2) Extraction of lung parenchyma with morphological reconstruction filtering

Although the target area of the lung parenchyma has been initially seen after the threshold segmentation of the original image, the background of the image window and the lung parenchyma are both low-density areas on the grayscale histogram, resulting in a false target area. Morphological reconstruction filtering can be regarded as a kind of nonlinear filtering. Unlike traditional nonlinear filtering, it is not simply a window function convolution operation based on the local characteristics of the image, but is divided into two processes: selection and reconstruction [10, 11]. The key to using morphological reconstruction filtering to extract lung parenchyma lies in how to generate suitable labeled images and construct corresponding filters. The specific algorithm steps are as follows:

Step 1. First, filter out the pseudo target area. Since the target area always touches the image boundary, the labeled image is defined as:

(9) $$\begin{array}{c} f=\left\{\begin{array}{cc} g\left(x,y\right), & \left(x,y\right)\text{ on the boundary of }g,\\ 0, & \text{other}, \end{array}\right.\\ w_{ij}=\frac{\left({tf}_{ij}\times \log\left(N/n_{i}\right)\right)}{\sqrt{\sum {\left[{tf}_{ij}\times \log\left(N/n_{i}\right)\right]}^{2}}}. \end{array}$$

Construct a pseudotarget area filter, and its function expression is *R*_*g*_(*f*)∩*g*. *f*_*ij*_ represents the frequency of *i* appearing in text *j*, *N* is the number of texts in *j*, and *n*_*i*_ is the number of texts where *i* appears.

RETRACTED

Step 2. To ensure the enforceability of subsequent processing, the extracted lung parenchyma needs to be filled with holes first, and the labeled image is defined as:

(10) $$\begin{array}{c} f=\left\{\begin{array}{cc} 1-g\left(x,y\right), & \left(x,y\right)\text{ on the boundary of }g,\\ 0, & \text{other}, \end{array}\right. \end{array}$$

(11) $$\begin{array}{c} w_{ij}=\frac{\left(\log\left({tf}_{ij}+1\right)\times \log\left(N/n_{i}\right)\right)}{\sqrt{\sum {\left[\log\left({tf}_{ij}+1\right)\times \log\left(N/n_{i}\right)\right]}^{2}}}. \end{array}$$

Thus, the lung cavity filling filter is constructed, and the function is expressed as [*R*_*g*^*C*^_(*f*)]^*C*^.

Step 3. Finally, remove irrelevant tissues such as trachea, effectively retaining the required lung parenchyma. Define the mark image as follows:

(12) $$\begin{array}{c} f=\left\{\begin{array}{cc} 1, & \left(x,y\right)\in \left\{P_{\text{left}},P_{\text{right}}\right\},\\ 0, & \text{other}, \end{array}\right. \end{array}$$

(13) $$\begin{array}{c} w_{ij}={tf}_{ij}\times {\left[\log\left[\overset{M}{\underset{i=1}{\sum }}\frac{{nt}_{i}}{{nt}_{i}}\right]\right]}^{2}. \end{array}$$

In the formula, *nt*_*i*_ represents the number of occurrences of *t*_*i*_ in the text, and *M* represents the total number of feature items. Use the middle row of the image matrix to calculate the number of target pixels appearing in each column on the left and right and divide the left and right columns by the middle column to find the maximum number of pixels [12]. The location of the maximum value is the seed point *P*_left_ of the left lung lobe and the seed point *P*_right_ of the right lung lobe. The reconstructed image *R*_*g*_(*f*) removes the atmospheric duct and some false target points remaining due to noise, and the lung parenchymal image is obtained initially.

(3) Left and right separation and edge repair of lung parenchyma

In the process of lung parenchymal segmentation, separation of left and right lungs and repair of the edges of lung regions are the links that need attention. The presence or absence of this process will directly affect the sensitivity and false positives of the subsequent detection of lung nodules [13]. In the middle and lower lung fields, it is difficult to avoid misclassification due to the threshold method, which leads to some depressions in the edge contour of the lung area. These depressions may be the growth location of pleural adhesions and lung nodules.

The lung parenchymal image is labeled using the run-length coding connected region labeling algorithm, and the label value is used to determine whether the left and right lungs are separated. If there is only one label value, the left and right lungs are in a connected state. At this time, the traversal space is limited to the lung area where the connecting run is located (usually in the upper lung area). Its upper and lower adjacent rows are in the interval between the travel distances. Find the maximum interval representing the left and right lung runs in the subimage, and replace the corresponding pixel values of the connected runs in the subimage with data bit alignment, so as to achieve the effect of separating the left and right lungs [14, 15].

RETRACTED

In the edge repair of lung parenchyma, firstly, the left and right lungs are tracked separately, and then, the lung parenchymal image is regarded as a partial two-dimensional convex hull, and the obtained edge points are corrected by the Graham scanning method. In the scanning process, it is necessary to limit the deflection angle and the distance of the correction line.

### 2.2. Suspected Nodule Enhancement Algorithm in the Lung Area

At present, most of the researches on enhancement algorithms for suspected nodules mostly use structural shape enhancement filtering methods. The specific principle is to use the second-order partial differential information of the image to establish the Hessian matrix and use different eigenvalues to have a strong response to different scales of spherical and linear structures and to construct filters to select nodules and blood vessels, respectively [16, 17]. However, this method has limitations: (1) the X-shaped or Y-shaped intersection of blood vessels cannot be effectively identified; (2) the target shape and structure selected by filtering are not completely accurate, especially for burrs, nodules; (3) since the Hessian matrix contains high-order partial differential information, the selected target may have false edges caused by noise points. In order to enhance the suspected lesion area to obtain a better effect, Gaussian smoothing filter is applied in a certain scale range, and then, a better nonlinear anisotropic diffusion filter-conversion tensor filter is implemented.

1. Gaussian smoothing preprocessing

The Gaussian kernel function has rotational symmetry, so the expression of the Gaussian kernel function in the two-dimensional case is:

(14) $$\begin{array}{c} G\left(x,y\right)=\frac{1}{\sqrt{2\pi \sigma }}e^{-\left(x^{2}+y^{2}\right)/2\sigma^{2}}. \end{array}$$

In Equation (11), *σ* is the scale parameter, which determines the smoothing effect of Gaussian filtering. On the other hand, it can be regarded as the recognition of the distance of the target in the visual psychology [18, 19]. As *σ* continues to increase, the target details of the image, such as the edge contour, become more and more blurred. Nonlinear anisotropic diffusion filtering allows the introduction of multiscale analysis. Since the size of the suspected nodules in the lung area is not fixed, multiscale analysis enables these suspected nodules of various sizes to be mapped into the scale space described by the Gaussian function. This scale space is usually measured by the scale parameter *σ*. Choose to perform Gaussian smoothing within a certain scale range, so that the gray unevenness that may appear in the suspected lesion area is eliminated, and the image quality is improved [20, 21].

(2) Conversion tensor filtering

Although the general tensor filtering can better enhance the structure of the corners and intersections in the image and even repair the discontinuous edges to a certain extent, however, the transform tensor filter cannot enhance the weak edge. Therefore, through in-depth analysis of the design of the diffusion tensor to make the tensor filtering play a better performance, so there are:

1. When *λ*1 ≈ *λ*2 ≈ 0, it means that the diffusion speed is very slow along any direction at this point of the image, corresponding to the uniform grayscale area of the image
2. When *λ*1 > >*λ*2 ≈ 0, it means that the diffusion speed at this point of the image along the vertical image characteristic direction is much larger than the image characteristic direction, corresponding to the edge of the image in the lungs
3. When *λ*1 ≈ *λ*2 > >0, it means that the diffusion speed along any direction at this point is quite fast, corresponding to the intersection of the linear regions in the image

In view of the above different situations, when the suspected nodule in the lung area is enhanced, the local consistency of the image is used to measure the local gray-scale contrast *H* = (*λ*1 − *λ*2)^2^ of the image. Obviously, this kind of local consistency can well describe various situations in the above image, such as *H* ≈ 0 when the gray level is uniform.

RETRACTED

Because a certain part of the boundary of the GGO nodule appears as a narrow boundary with a low contrast of grayscale changes, the corresponding first-order derivative has a small value, even close to zero. This shows that the image gradient modulus is difficult to accurately describe the weak boundary. However, the weak boundary correspondence is reflected as an extreme value on the second-order directional derivative of the image, so the Hessian matrix of the image should be able to reflect the weak boundary information well [22, 23]. In order to better understand the first-order partial differential information in the gradient, a conversion structure tensor with autocorrelation and cross-correlation characteristics is used to automatically select two different structure tensors according to the edge information (gradient modulus) of the image. The amount:

(15) $$\begin{array}{c} J=\left\{\begin{array}{cc} J_{H} & \left|\nabla u_{\sigma }\right|<T,\\ \rho & \left|\nabla u_{\sigma }\right|\geq T. \end{array}\right. \end{array}$$

In Equation (12), *T* is the threshold parameter of the gradient modulus, and the diffusion tensors corresponding to *J*_*H*_ and *J*_*ρ*_ are *D*_*H*_ and *D*_*ρ*_, respectively. The diffusion tensor is derived from the structure tensor, and the eigenvectors and eigenvalues of the diffusion tensor, respectively, correspond to the consistency direction and metric information. *D*_*H*_ is the Hessian matrix, and the eigenvalues *λ*1 and *λ*2 in the diffusion tensor *D*_*ρ*_ are designed as follows:

(16) $$\begin{array}{c} \begin{array}{c} \lambda 1=c,\\ \lambda 2=\left\{\begin{array}{c} c,\mu 1=\mu 2,\\ c+{\left(1-c\right)}^{\beta /{\left(\mu 1-\mu 2\right)}^{2}},\text{other}. \end{array}\right. \end{array} \end{array}$$

In formula (13), *μ*1 and *μ*2 are the eigenvalues corresponding to the structure tensor *J*_*ρ*_, the parameter *c* is usually a small decimal, and *β* is the consistency parameter of *μ*1 and *μ*2 [24, 25]. By setting the parameters of Equation (13), the diffusion process continues in the consistent direction, smoothing the uneven area, effectively suppressing the vertical direction, and retaining boundary information.

RETRACTED

## 3. Experimental Design of Auxiliary Diagnosis System for Chest CT Assessment of Pulmonary Nodules

### 3.1. Tools Required for System Development

1. VTK

VTK provides cross-platform development, supports multiple operating systems, and also supports algorithms such as vectors, vectors, tensors, and textures. As medical technology has higher and higher requirements for visualization, VTK has more and more extensive applications in medical image visualization by virtue of its advantages in this regard.

(2) ITK

ITK is customer-oriented, it can be connected across platforms, and it can provide very accurate algorithmic calculations on image segmentation, but its advantages are more than that.

(3) Combination of ITK and VTK

ITK and VTK have their own focus. Therefore, combining ITK with VTK and complementing each other will solve the problem that ITK has powerful data processing functions, but it has the disadvantage that it cannot be monitored at any time, while VTK does not have powerful data processing functions.

### 3.2. System Function Design

By learning the process of radiologists diagnosing pulmonary nodules, the pulmonary nodule diagnosis CAD system is mainly divided into four steps. The first step is to segment the lung and find the lung accurately in the chest CT image; the second step is to detect suspicious pulmonary nodules in the segmented lung; the third step is the image feature extraction process of suspicious pulmonary nodules as the basis for further analysis; the fourth step is to identify the suspicious pulmonary nodules and judge whether the pulmonary nodules are benign or malignant through the early extracted features. In general, it is to determine the lung detection area first, use CT images to detect whether there are suspicious pulmonary nodules, and judge the benign and malignant of pulmonary nodules. For a complete auxiliary diagnosis system, in addition to these four diagnostic processes, it should also include the reading and analysis of CT images, the display of images, and the marking of pulmonary nodules, so that doctors can mark the discovered pulmonary nodules for and auxiliary diagnosis. The system function design of the system is shown in Figure 3.

RETRACTED

As shown in Figure 3, they are the reading of CT images, the segmentation of lung regions, the detection of suspicious lung shadows, the feature extraction of suspicious lung shadows, the identification of suspicious lung shadow properties, the display of CT images, and the marking of suspicious lung nodules. And interact. The four parts in the middle are the key to the system, and the effect of each part affects the performance of the entire system.

### 3.3. Experimental Objects and Experimental Methods

In this paper, CT images of patients' lungs are selected as the detection objects of the auxiliary diagnosis system, and there are 8 groups in total. The detailed information of each patient's CT image is shown in Table 1. The number of CT images is different for different patients and equipment manufacturers; pixel pitch and slice distance are also different. The system first reads the three-dimensional image of the patient and then segmentation of the lung area. The segmented lungs are detected with a variable loop filter to detect suspected shadows, and then, the feature values of the detected shadows are calculated, and finally, the suspected shadows are calculated by the classifier. The shadows are classified to complete the entire auxiliary diagnosis process of lung nodules. The number of nodules, the number of malignant nodules, and the number of false positives of each set of lung CT images were obtained to analyze the performance of the auxiliary diagnosis system.

## 4. Experimental Auxiliary Diagnosis System for Chest CT Assessment of Pulmonary Nodules

### 4.1. Classifier ROC Curve Analysis

The classifier is tested using the training data of lung nodules. The data contains 390 training data, including 219 benign samples, 171 malignant samples, and 179 test data, including 41 benign samples and 138 malignant samples. According to the possibility that benign shadows may be blood vessels perpendicular to the slice, benign nodules, etc., the number of clusters of benign shadows is selected between 4 and 8. According to the possibility that the malignant shadow may be a solitary pulmonary nodule, semisolitary pulmonary nodule, ground glass shadow, etc., the number of malignant shadow clusters is selected between 3 and 6. The number of clusters is determined by interleaving the training data, the number of benign shadow clusters is 5, and the number of malignant shadow clusters is 4, and then, the test data is used for testing. The ROC curve of the test results is shown in Figure 4.

RETRACTED

It can be seen from Figure 4 that the sensitivity of the classifier based on fuzzy clustering and Mahalanobis distance rises rapidly at the beginning of the curve, when the value is 0.2, the sensitivity of the classifier based on fuzzy clustering and Markov distance reaches the highest point and tends to be stable, and the area under the curve is much larger than the area of the ROC curve of the Fisher linear classifier. The classifier based on fuzzy clustering and Mahalanobis distance can classify the data better than the Fisher linear classifier.

### 4.2. Image Display Module Implementation

After the image is read in, it must be displayed in time for the user to read. Define a pointer of the vtkImageData class in the document class to save the vtk image. Complete the conversion from ITK data to VTK data through the ITKtoVTKImageFilter class, and then, use the vtkImageFlip class to flip the converted image into the *y*-axis to realize the conversion from the ITK coordinate system to the VTK coordinate system. After getting the VTK data, the document uses UpdateAllViews() to update all the views. Since the resolution of the CT image is much higher than that of the human eye, in order to map the read image to the window width and window level of the image to be read in a range suitable for reading, the reading flow chart is shown in Figure 5.

After obtaining the appropriate window width and window level, the VTK image data pixels are mapped to the appropriate range through the mapping of vtkMapper. For two-dimensional images, after converting the data into vtkActor, it can be added to the vtkRenderer class for display. The two-dimensional DICOM image display is shown in Figure 6.

For three-dimensional images, in order to allow physicians to obtain more image information and make better judgments, three-dimensional cross-sectional views can be displayed. At this time, three vtkActors are needed, and each vtkActor displays a section. Setting the display range of each vtkActor can achieve the same position as the section in the three-dimensional image. The three-section display of a three-dimensional image is achieved through the combination of three sections. Adding an interactive device to the view can realize the interaction between the mouse and the image, such as zooming and rotating. The three-dimensional cross-sectional view is shown in Figure 7.

RETRACTED

The vtkImageReslice class in the VTK development kit can extract any section of a three-dimensional image by setting the origin and normal vector. If the origin is set at the center of the three-dimensional image and the normal vectors are in the *z*-axis direction, *x*-axis direction, and *y*-axis direction, respectively, a cross section, sagittal plane and coronal plane passing through the image center can be obtained (as shown in Figure 8).

### 4.3. Implementation of Lung Segmentation Module

This module realizes segmentation of the lung area in the image. Since a set of CT images consists of more than 300 images, each image has a resolution of 512 × 512. It takes a long time to traverse the image multiple times. At the same time, medical images have a lot of noise due to errors in the *X*-signal acquisition equipment. Therefore, it is necessary to denoise the image. In order to improve the contrast sensitivity of the image and display the fuzzy and poor contrast details in the image, it is also necessary to enhance the image. The result of binarization of the original image is shown in Figure 9(a).

So, the linear interpolation method is used to down-sample each layer of the original image, and the sampling rate is 1 : 2. Since the density of human tissue is gradual to a large extent, and most medical images also show gradual characteristics, it is more appropriate to use linear interpolation whether to enlarge, reduce, or rotate the medical image. The number of image layers after sampling remains the same, but the resolution of each image is reduced to 256 × 256, and the data volume is reduced to a quarter of the original. At the same time, the image is also smoothed to reduce the impact of noise, but the boundary of the image still clear (as shown in Figure 9(b)).

Next, the optimal threshold method is used to obtain the optimal segmentation threshold *T* to binarize the image. The pixels smaller than the threshold *T* become white, and the threshold larger than the threshold *T* becomes black (as shown in Figure 10(a)). In the binarized image, the white area is equivalent to the foreground (object), and the black area is equivalent to the background. Then, the foreground area in the three-dimensional medical image is marked using the method of three-dimensional area connection marking. We think that the foreground area that is adjacent to the image boundary is the empty area surrounding the body. By traversing the four boundaries of each layer of the entire three-dimensional image, the labels of all the foreground areas that are adjacent to the boundary can be obtained. Except for the foreground area of the air area, the lung area should be the largest area. By counting the number of pixels in each foreground area except the air area, the two areas that are the largest and greater than a certain threshold are reserved as the lung area. Through experiments, we take one percent of this threshold. The resulting lung area is shown in Figure 10(b).

RETRACTED

At this time, the lung area is full of cavities, and the edges are not smooth, which cannot meet the requirements for segmenting the lung area. Next, use the hole filling algorithm of geodesic distance to fill the lung area (as shown in Figure 11(a)). For the filling algorithm of the deformed median filter algorithm, the determination of the radius *r* of the neighborhood, the threshold *T*, and the number of iterations *N* is the key to whether the algorithm can achieve the predetermined effect. If the neighborhood radius *r* and the number of iterations *N* are too small, it is difficult to fill large depressions such as the hilum; if the neighborhood radius and the number of iterations are too large, the calculation time will be too long. Threshold is too small, it will not work for depressions with small arcs. Threshold is too large; it will fill the contour of the normal lung. Through a large number of experiments, it is found that when the radius *r* is set to 5, the threshold *T* is set to 8, and the number of iterations *N* is set to 8, the repair effect is better, as shown in Figure 11(b), and the ability to oversampling also reduces the amount of calculation and increases the speed.

The repaired image is enlarged to the size of the original image by the nearest neighbor interpolation method, and this is used as a mask to segment the lung image as shown in Figure 12. The segmentation effect is better.

### 4.4. System Test Results

The system goes through the entire lung nodule auxiliary diagnosis process, and the specific situation is shown in Table 2.

As can be seen from Table 2, the above images have a total of 2316 CT images and 56 nodules. A total of 49 nodules were detected, and 7 were missed. A total of 64 false-positive nodules were detected, with an average of 8 per image. The layer distance images are all valid, and the overall sensitivity is high, which can effectively provide doctors with advice.

## 5. Conclusions

This paper constructs a complete computer-aided diagnosis system, which includes 7 modules including lung suspicious shadow detection, lung suspicious shadow property judgment, and CT image display. This article not only uses the original ROI as the feature extraction object but also adds two enhanced ROIs as the feature extraction object. For these three types of ROI, features based on geometric shapes, features based on gray information, features based on boundary radiation, and features based on location information are extracted, respectively. The system detected 56 nodules in CT images, 49 were actually detected, 7 were missed, and the detection rate was 87.5%, with an average of 8 false-positive nodules per set of images. Experiments have proved that the system has good effects on CT images of different equipment, pixel pitch, and slice pitch and has high sensitivity, which can provide doctors with good advice. Disadvantages of this article: high false-positive rate. This problem exists mainly because the characteristics of different nodules are very different. The threshold must be lowered, which increases the probability of detecting false-positive nodules. Computer-aided diagnosis is an important development direction of imaging diagnostics. At present, the performance of pulmonary nodule-aided diagnosis system needs to be improved. Increasing the false-positive rate while improving the detection rate has become an important factor restricting its wide application. How to make full use of image data, combined with medical anatomy and diagnostic knowledge, improve the detection rate of computer-aided diagnosis and reduce its false-positive rate which has become the focus and hotspot of future research.

RETRACTED

## Figures and Tables

**Figure 1:** Chest CT image and gray histogram analysis.

**Figure 2:** Threshold classifier and threshold segmentation results.

**Figure 3:** Functional design of auxiliary diagnosis system for pulmonary nodules.

**Figure 4:** ROC curve of classifier.

**Figure 5:** Flow chart for reading window width.

**Figure 6:** Display diagram of two-dimensional image.

**Figure 7:** Three-dimensional cross-sectional view rotated at a certain angle.

**Figure 8:** Sectional view of three-dimensional image in three directions.

**Figure 9:** Binarization and down-sampling CT images.

**Figure 10:** Binarization and retained lung area map after downsampling.

**Figure 11:** Lung area before and after filling.

**Figure 12:** Segmented lung image.

**Table 1:** Patient image information sheet.

Numbering	Number of images	Equipment manufactory	Pixel pitch (mm)	Layer distance (mm)	Number of nodules (*a*)
1	336	Philips	0.68	1	5
2	277	Philips	0.60	1	3
3	266	GE	0.76	1.25	12
4	290	GE	0.71	1.25	1
5	249	GE	0.62	1.25	7
6	233	Philips	0.60	1	2
7	247	GE	0.60	1.25	24
8	429	Philips	0.68	1.5	2

**Table 2:** Patient image information sheet.

Patient		Variable loop filter test results		Classifier classification results	
Numbering	Number of nodules	Malignant nodules	Number of false positives	Malignant nodules	Number of false positives
1	5	5	121	5	10
2	3	3	83	3	5
3	12	10	114	10	7
4	1	1	137	1	7
5	7	6	169	6	8
6	2	2	153	2	8
7	24	21	134	20	12
8	2	2	197	2	7
Total	56	50	1108	49	64

RETRACTED

## Data Availability

We do not have permission to share data from the data provider.
